The article "Efficacy of NHP66 Bioactive Cage on Patients with Cervical Spine Injury in Short-Track Speed Skating" was retracted in 2023. Reasons: unreliable results or conclusions; lack of ethics approval or compliance; concerns about the data; concerns about the peer review.

# Efficacy of NHP66 Bioactive Cage on Patients with Cervical Spine Injury in Short-Track Speed Skating

**DOI:** 10.1155/2022/6088398

**Published:** 2022-01-29

**Authors:** Xinming Yang, Fei Liu, Yanlin Yin, Peinan Zhang, Yongli Jia, Ying Zhang, Yao Yao, Ye Tian

**Affiliations:** ^1^Department of Orthopaedics, The First Affiliated Hospital of Hebei North University, Zhangjiakou, 075000 Hebei, China; ^2^Department of Orthopaedics, The First Hospital Of QinHuangDao, Qinhuangdao City, 066000 Hebei, China

## Abstract

**Background:**

Short-track speed skating (STSS) is an extreme sport in pursuit of extreme speed and explosive force. In such a sport, once athletes fall down, they are susceptible to serious cervical spine injury (CSI) under the inertia of high-velocity movement. Nanohydroxyapatite/polyamide 66 (NHP66) bioactive cage is a high-tech product of nanotechnology in the medical field in recent years. With a structure similar to that of human cortical bone, NHP66 bioactive cage has extremely high toughness and strength, which tailors to the needs of STSS.

**Objective:**

This study mainly analyzed the therapeutic effect of NHP66 on patients with CSI in STSS, aiming to provide new opportunities for the treatment of this patient population.

**Methods:**

A total of 51 patients with CSI treated in our hospital were enrolled, including 19 cases of short-track speed skaters (observation group) and 32 cases of car accidents, falls from heights, or collision injuries (control group). The relevant surgical indicators (operation time, intraoperative blood loss, etc.), the incidence of adverse reactions, the Cobb angle of cervical lordosis before and after surgery, and the fusion segment height of the cage were observed and compared between the two groups. Postoperative pain was evaluated by the visual analog scale (VAS), improvement of spinal cord injury was assessed by the American Spinal Cord Injury Association (ASIA) Impairment Scale, and bone fusion, bone subsidence, and other motor functions were assessed by the Japanese Orthopaedic Association (JOA) score rating system.

**Results:**

The operation time, intraoperative blood loss, and incidence of adverse reactions in the observation group were significantly lower than those in the control group. The Cobb angle of cervical lordosis and the fusion segment height of cage increased significantly higher in both groups after surgery. In addition, the VAS scores of the observation group 2 h and 3 d after operation were significantly lower than those of the control group. In terms of improvement of spinal cord injury, ASIA and JOA scores in the observation group were significantly higher than those before treatment and in the control group. There was no significant difference in bone fusion activity between the two groups.

**Conclusions:**

In this study, it is found through experiments that NHP66 has higher safety and application value than autogenous iliac bone, confirming that NHP66 can achieve significant results as a cage for anterior cervical decompression and iliac bone graft fusion and internal fixation in short-track speed skaters after CSI.

## 1. Introduction

In the fierce and fast movements of competitive sports, athletes are susceptible to injuries due to accidents [1]. Short-track speed skating (STSS) is an extreme sport in pursuit of extreme speed and explosive force. In such a sport, once falling or wrestling due to improper operation, athletes are prone to serious injuries under the inertia of high-velocity movement, among which cervical spine injury (CSI) is a common one [2, 3]. According to relevant data, the risk of serious CSI in STSS is as high as 10%-20% [4]. CSI, often accompanied by varying degrees of dystonia and pathological reflex that result in motor, sensation, and sphincter dysfunction, may even cause disability and paralysis in athletes due to nerve compression in severe cases [5]. Therefore, the management of CSI requires extreme caution, and a complete cure is of particular importance for athletes because of its potential disruption to their careers [6].

Currently, conservative treatment is reserved for patients with mild CSI, while surgery is indicated for those with severe CSI combined with spinal cord injury (SCI) [7]. Anterior cervical decompression (ACF) combined with iliac bone graft fusion and internal fixation is commonly used in the treatment of severe CSI, which can fully decompress the cervical spinal canal under direct vision and repair and reconstruct the damaged anterior column of the cervical spine [8]. The prognosis of patients depends largely on the choice of materials for anterior cervical cage [9]. Autologous iliac bone (AIB), with a clinically recognized bone fusion rate, is the most commonly used material for reconstruction [10]. However, AIB is not suitable for short-track speed skaters who need to perform high-intensity training and exercise after rehabilitation due to its low strength to provide insufficient support, inclination to absorption and subsidence, and the risk of infection at the donor site [11]. Therefore, the key to solving CSI of competitive athletes is to find a reconstruction material for bone cage with better osteoconductivity and mechanical properties.

Nanohydroxyapatite/polyamide 66 (NHP66) bioactive cage, as a high-tech product with increasingly mature applications of nanotechnology in the medical field in recent years, has achieved remarkable achievements in decompression and fusion for cervical spondylosis [12]. NHP66 has a similar structure to human cortical bone, with marvelous toughness, stress strength, and fusion with bone [13]. Studies have shown that NHP66 can also form an antibacterial and anti-inflammatory biological scaffold with antimicrobial titanium, which has a certain adjuvant therapeutic effect on infected bone defects or osteomyelitis [14]. For short-track speed skaters, they need not only to restore the height of the injured vertebrae and reconstruct the normal sequence of cervical vertebrae but also more stable internal fixation and a higher rate of intervertebral fusion. And this is where NHP66 comes in. Therefore, this study analyzed the efficacy of NHP66 on patients with CSI in STSS, with the aim of providing reliable theoretical guidance for patients with CSI in competitive sports in the future.

## 2. Materials and Methods

### 2.1. General Data

A total of 51 patients with CSI admitted to our hospital between May 2018 and April 2020 were enrolled. Among them, 19 STSS athletes were assigned to an observation group, and the other 32 patients injured due to traffic accident, falls from heights, or collision injuries were included in a control group. This study, approved by the Ethics Committee, was conducted in strict accordance with the Declaration of Helsinki. The subjects were fully informed of the purpose of the study and submitted an informed consent.

### 2.2. Inclusion and Exclusion Criteria

Inclusion criteria: patients (20-40 years old) who were confirmed with cervical vertebra fracture by X-ray, CT, and MRI, with the presence of intervertebral height decrease, segmental kyphosis, cervical cord compression by fracture or ruptured cervical tissue, and vertebral subluxation, were enrolled. Exclusion criteria: patients with other cardiocerebrovascular diseases, congenital abnormality of cervical spine, cervical locked facet, or allergies to drugs used in this study were excluded, as well as referrals.

### 2.3. Surgery Methods

The patient was placed in a supine position with the neck naturally tilted back under routine intratracheal intubation anesthesia. An anterior transverse incision was made based on the level of the injured vertebra, and blunt dissection was performed along the gap of loose connective tissue between the cervical visceral sheath and the carotid sheath. Then, the injured vertebra was located by X-ray. Subsequently, corpectomy of the injured vertebra was performed. The spinal canal was decompressed thoroughly, and the intervertebral space was distracted to restore the physiological curvature of cervical lordosis, so as to measure the height of intervertebral groove. For patients in the observation group, NHP66 bioactive cage was used as the vertebral cage, and the bone fragments dropping during spinal canal decompression were filled into the hollow part of the cage and implanted into the intervertebral bone groove. For patients in the control group, AIB was used as a cage. An oblique incision of about 4 cm long was made on the patient's right iliac crest, and a full plate iliac bone strip of about 1.5 × 3.5 cm in size was cut with an osteotome and implanted into the intervertebral bone groove. After implantation, the distractor was released, followed by appropriate compression, anterior cervical titanium plate internal fixation, drainage tube placement, and incision suture. After surgery, patients in both groups were given hormones, dehydrants, antibiotics, and neurotrophic drugs. In addition, they wore a neck brace for 3 months, and the stitches were removed on the 7th day after surgery.

### 2.4. Outcome Measures

Clinical baseline data of patients in the two groups: surgical indicators: intraoperative blood loss and operation time were recorded in both groups. Safety: the incidence of adverse reactions after surgery was calculated in both groups. The cage: lateral cervical spine X-ray examination and CT scan were performed before surgery and 7 days after surgery, and the fusion segment height of the cage and the Cobb angle of cervical lordosis were measured. Pain: the visual analog scale (VAS), with a score ranging from 0 to 10, was used to evaluate the pain of patients at 2 h and 3 d after surgery; the score is proportional to the degree of pain. Alleviation of SCI: before surgery and 7 days after surgery, each patient was assessed for the degree of SCI according to SCI grading criteria developed by the American Spinal Injury Association (ASIA); on a 100-point scale, the score was in inverse proportion to the degree of injury. Bone fusion: the fusion of the implanted bone in the two groups was reexamined at 6 months after surgery. Once the implanted bone was fused, all the interfaces between the implant and the adjacent vertebral endplates became blurred, and new continuous bone trabeculae could be seen passing through the cage and the upper and lower endplates. The change of fusion segment height ≥ 3 mm was judged as subsidence. Motor function: the Japanese Orthopaedic Association (JOA) score rating system, with a score ranging from 0 to 17 points, was used to assess the improvement of cervical function of patients before surgery and at 6 months after surgery; the lower the score, the more obvious the spinal dysfunction. Characterization and observation of NHP66: NHP66 tissues were ground into powder and added into a proper amount of normal saline. The powder sample was then observed under a microscope, and the particle size and potential of nanoparticles were evaluated with a potentiometer.

### 2.5. Statistical Analysis

All data in this study were analyzed by SPSS25.0. Counting data, such as sex, residential environment, and injury site, were recorded in the form (*n* (%)) and analyzed using the chi-square test. Measurement data, such as age and body mass index (BMI), were expressed as ($\bar{\chi }\pm s$), and the intergroup and intragroup comparisons before and after therapy were performed by the independent-samples *t*-test and paired *t*-test, respectively. *P* < 0.05 indicated a statistically significant difference.

## 3. Results and Discussion

### 3.1. Clinical Baseline Data

The two groups were not significantly different in age, sex, BMI, residential environment, injury site, CSI grade, exercise habit, and ethnicity (all *P* > 0.05, Table 1).

### 3.2. Surgical Indicators

The intraoperative blood loss and operation time were compared between the two groups. It was found that the operation time (min) of the observation group was significantly shorter than that of the control group (94.21 ± 7.45 vs. 138.36 ± 8.57, *P* < 0.05), and the intraoperative blood loss (mL) was significantly less in the observation group compared with the control group (140.12 ± 28.45 vs. 181.39 ± 37.67, *P* < 0.05) (Figure 1).

### 3.3. Incidence of Postoperative Adverse Reactions

The observation group showed a total incidence of postoperative adverse reactions of 15.79%, including 0 cases of infection, 1 case of pain, and 2 cases of numbness, while the control group showed a total incidence of 43.75%, including 4 cases of infection, 5 cases of pain, and 5 cases of numbness. The incidence of postoperative adverse reactions in the observation group was significantly lower than that in the control group (*P* < 0.05, Table 2).

### 3.4. Cage Analysis

Lateral cervical spine X-ray examination and CT scan were performed before and 7 days after surgery, and the fusion segment height and Cobb angle of cervical lordosis were analyzed. The results showed that the fusion segment height and Cobb angle of cervical lordosis were not significantly different between the two groups before surgery (*P* < 0.05), while increased greatly in both groups after surgery (*P* < 0.05, Figure 2).

### 3.5. Postoperative Pain

The pain of patients in the two groups was evaluated using the VAS at 2 h and 3 d after surgery. The results showed that the VAS score in the observation group was significantly lower than that in the control group both at 2 h and 3 d after surgery (*P* < 0.05, Figure 3).

### 3.6. Alleviation of SCI and Improvement of Motor Function

The alleviation of SCI and improvement of motor function of the two groups were evaluated by the SCI grading criteria developed by the ASIA and the JOA score rating system before surgery and at 6 months after surgery, respectively. The results showed that there were no statistically significant differences in ASIA and JOA scores before surgery (*P* > 0.05); after surgery, the ASIA and JOA scores of both groups increased and the scores of the observation group were higher than those of the control group (both *P* < 0.05, Figure 4).

### 3.7. Movement Function

In the observation group, all patients had successful bone fusion, while in the control group, 93.75% of patients had bone fusion and 6.25% of them had bone subsidence. Nonetheless, there was no statistical difference in bone fusion between the two groups (*P* > 0.05, Table 3).

### 3.8. Characterization and Observation of NHP66

Microscopically, NHP66 had an extremely dense and evenly distributed molecular structure, with a very small internanoparticle gap and particle size of about 150 nm. As determined by a potentiometer, the zeta potential and PDI of NHP66 were approximately 3.26 and 0.36, respectively (Figure 5).

## 4. Discussion

In addition to the serious trauma of bone tissue, the fracture fragments and broken cervical intervertebral disc tissue generated in CSI may compress and stimulate the spinal cord, leading to neurological dysfunction [15]. Therefore, the treatment principle for SCI is to completely decompress the spinal canal and reconstruct the anterior column of the cervical spine, so as to restore the normal sequence and stability of the cervical spine and avoid nerve injury [16, 17]. ACF combined with iliac bone graft fusion and internal fixation is the first choice for CSI, and its effectiveness has been repeatedly confirmed clinically [18, 19]. The anterior cervical approach allows full decompression of the spinal canal under direct vision, which facilitates the reconstruction of damaged cervical vertebrae [20]. AIB is one common choice for reconstruction of the anterior column, with high safety and remarkable fusion rate [21]. However, the ilium, as a cancellous bone with thin cortical bone, has low strength and is prone to subsidence and collapse [22]. For STSS athletes, the strength of the cage is of particular importance for adaption to fierce sports confrontation [23]. Additionally, the integrity of lower limbs is crucial for STSS, as the sport requires strong explosive power of legs. In light of the above reasons, AIB is not suitable for restoring CSI in STSS athletes. The cage for the anterior column of the spine must have favorable biocompatibility, high toughness, and mechanical properties, with the ability to effectively induce osteoblast activity and facilitate clinical examination [23]. NHP66 is an optimal material able to perfectly meet the above requirements. As a coprecipitation product of hydroxyapatite and polyamide 66, NHP66 has a similar structure to collagen, without toxic or side effects on the human body [24]. And in virtue of the dense nanomolecular structure, NHP66 boasts of fabulously high toughness and excellent compatibility with tissues [25]. In one earlier study [26], NHP66 has served as an ideal fusion device for spinal anterior reconstruction, effectively restoring and maintaining spinal alignment and intervertebral height. NHP66 is of greater value for STSS athletes.

In our study, we compared NHP66 with AIB in various aspects. First, we found that patients in the observation group treated by NHP66 experienced shorter operation time and less intraoperative blood loss than those in the control group treated by the ilium, which is consistent with our expectations. Patients treated with iliac bone as cage required not only cervical vertebra surgery but also additional removal of the iliac bone, so they experienced longer operation time and more blood loss than those in the observation group requiring only cervical vertebra surgery. Then, we calculated the incidence of postoperative adverse reactions in the two groups and found a significantly lower incidence in the observation group compared with the control group. The results suggest that NHP66 may be safer than AIB, and the reason behind it, we speculate, may be related to the shorter operation time and less blood loss in this procedure. In a long-term operation, the patients' internal environment and tissues are exposed for a longer time, which increases the possibility of oxidative stress and inflammatory reaction and consequently elevated risk of postoperative infection and pain. Subsequently, we compared the condition of the cage in the two groups. The results showed that the intervertebral height and Cobb angle of the cervical fusion segment of both groups were improved after surgery, with no significant difference between the two groups, suggesting the excellent improvement effects of both NHP66 and ilium. However, the observation group experienced better alleviation of postoperative pain and injury than the control group. In addition, all patients in the observation group had bone fusion, but some in the control group had bone subsidence. The results might be caused by the excessive curettage of adjacent vertebral bone endplate during surgery. Moreover, with a small and dense molecular structure, NHP66 can closely contact intervertebral nerve and muscle tissue and act as an annular cage, thus reducing the friction against endplate. After implantation, the molecular structure of NHP66 can slowly change to a height and curvature suitable for the cervical vertebra, and the nanomolecular particles can effectively adsorb osteoblasts, further improving the stability.

The novelty of this study lies in the evaluation of clinical advantages of NHP66 bioactive cage in short-track speed skaters from multiple dimensions including surgical indicators, safety, cage, pain, alleviation of spinal cord injury, and improvement of motor function, providing a new effective treatment strategy for short-track speed skaters with CSI. However, due to the short experimental period, the prognosis of athletes implanted with NHP66, one crucial index for the evaluation of NHP66, has not been followed up. We will follow up all participants of this study for a longer time to improve our results.

## 5. Conclusion

With excellent mechanical strength and toughness, NHP66 can deliver remarkable results as a cage for ACF combined with iliac bone graft fusion and internal fixation for athletes with CSI in STSS.

## Figures and Tables

**Figure 1:** Surgical indicators of the two groups: (a) operation time of the two groups; (b) intraoperative bleeding of the two groups. ^∗^*P* < 0.05.

**Figure 2:** Analysis of the cage of the two groups: (a) preoperative and postoperative Cobb angle of cervical lordosis in the two groups; (b) preoperative and postoperative fusion segment height of the two groups. ^∗^*P* < 0.05.

**Figure 3:** Postoperative pain of the two groups. ^∗^*P* < 0.05.

**Figure 4:** Alleviation of SCI and improvement of motor function: (a) ASIA score of the two groups; (b) JOA score of the two groups. ^∗^*P* < 0.05.

**Figure 5:** Characterization and observation of NHP66: (a) NHP66 under a microscope; (b) zeta potential and PDI of NHP66.

**Table 1:** General data (*n* (%)).

	Observation group (*n* = 19)	Control group (*n* = 32)	*t* or *χ*^2^	*P*
Age (Y)			1.211	0.232
	35.7 ± 3.2	34.6 ± 3.1		
Sex			0.158	0.691
Male	10 (52.63)	15 (46.88)		
Female	9 (47.37)	17 (53.13)		
BMI (kg/cm^2^)			0.406	0.687
	23.62 ± 2.18	23.36 ± 2.23		
Residential environment			1.893	0.169
Urban area	19 (100.00)	29 (90.63)		
Rural area	0 (0.00)	3 (9.38)		
Injury site			0.138	0.709
Upper cervical vertebra	14 (73.68)	22 (68.75)		
Lower cervical vertebra	5 (26.32)	10 (31.25)		
Upper and lower cervical vertebrae				
CSI grade			0.051	0.997
A	3 (15.79)	5 (15.63)		
B	6 (31.58)	11 (34.38)		
C	8 (42.11)	13 (40.63)		
D	2 (10.53)	3 (9.38)		
Exercise habit			3.291	0.070
Yes	19 (100.00)	27 (84.38)		
No	0 (0.00)	5 (15.63)		
Ethnicity			0.021	0.885
Han	18 (94.74)	30 (93.75)		
Ethnic minorities	1 (5.26)	2 (6.25)		

**Table 2:** Comparison of the incidence of postoperative adverse reactions between two groups (*n* (%)).

	Observation group (*n* = 19)	Control group (*n* = 32)	*χ* ^2^	*P*
Infection	0 (0.00)	4 (12.50)		
Pain	1 (5.26)	5 (15.63)		
Numbness	2 (10.53)	5 (15.63)		
Incidence of complications (%)			4.194	0.041
	15.79	43.75		

**Table 3:** Bone fusion.

	Observation group (*n* = 19)	Control group (*n* = 32)	*χ* ^2^	*P*
Fusion rate	19 (100.0)	30 (93.75)	1.236	0.266
Subsidence (≥3 mm)	0 (0.00)	2 (6.25)		

## Data Availability

The labeled dataset used to support the findings of this study is available from the corresponding author upon request.

## References

[1] Jederstrom M., Agnafors S., Ekegren C. (2021). Determinants of sports injury in young female Swedish competitive figure skaters. *Frontiers in Sports and Active Living*.

[2] Alas H., Pierce K. E., Brown A. (2021). Sports-related cervical spine fracture and spinal cord injury: a review of nationwide pediatric trends. *Spine*.

[3] Swiatek P. R., Nandurkar T. S., Maroon J. C. (2021). Return to play guidelines after cervical spine injuries in American football athletes: a literature-based review. *Spine*.

[4] Leider J., Piche J. D., Khan M., Aleem I. (2021). Return-to-play outcomes in elite athletes after cervical spine surgery: a systematic review. *Sports Health*.

[5] Keidan L., Barash A., Lenzner Z., Pick C. G., Been E. (2021). Sexual dimorphism of the posterior cervical spine muscle attachments. *Journal of Anatomy*.

[6] Schroeder G. D., Canseco J. A., Patel P. D. (2020). Updated return-to-play recommendations for collision athletes after cervical spine injury: a modified Delphi consensus study with the cervical spine research society. *Neurosurgery*.

[7] Liu Z., Li W., Xu Z. (2020). Treatment of monosegment spinal tuberculosis via posterior unilateral vertebral lamina fenestration debridement and bone grafting fusion combined with laminar reconstruction and internal fixation: a retrospective case- control study with a minimum 5-year follow-up. *World Neurosurgery*.

[8] Atinga M., Gregor R., Selvaraj K. M., Hong T. F. (2018). Os acromiale open reduction and internal fixation: a review of iliac crest autogenous bone grafting and local bone grafting. *Journal of Shoulder and Elbow Surgery*.

[9] Pojskic M., Saβ B., Nimsky C., Carl B. (2020). Application of an expandable cage for reconstruction of the cervical spine in a consecutive series of eighty-six patients. *Medicina*.

[10] Wu S., Lin B., Li X. (2021). Single-stage debridement via autogenous iliac bone graft through the olif corridor and lateral fixation in treating spontaneous single-level lumbar pyogenic spondylodiscitis. *BMC Musculoskeletal Disorders*.

[11] Hu J., Ou Y., Zhu Y. (2019). Effectiveness of nano-hydroxyapatite/polyamide-66 cage in interbody fusion for degenerative lumbar scoliosis. *Zhongguo Xiu Fu Chong Jian Wai Ke Za Zhi*.

[12] Zhao W., He B., Zhou A. (2019). D-rada16-rgd-reinforced nano-hydroxyapatite/polyamide 66 ternary biomaterial for bone formation. *Tissue Engineering and Regenerative Medicine*.

[13] Zhong W., Liang X., Luo X., Quan Z., Jiang D. (2020). Imaging evaluation of nano-hydroxyapatite/polyamide 66 strut in cervical construction after 1-level corpectomy: a retrospective study of 520 patients. *European Journal of Medical Research*.

[14] Zavvarian M. M., Hong J., Khazaei M. (2021). The protein kinase inhibitor midostaurin improves functional neurological recovery and attenuates inflammatory changes following traumatic cervical spinal cord injury. *Biomolecules*.

[15] Chilvers G., Janjua U., Choudhary S. (2017). Blunt cervical spine injury in adult polytrauma: incidence, injury patterns and predictors of significant ligament injury on ct. *Clinical Radiology*.

[16] Xie T., Feng Y., Song J., Yao G. (2021). Anterior dorsal root entry zone approach in the treatment of spinal intramedullary glioma. *World Neurosurgery*.

[17] Shaaya E., Fridley J., Barber S. M. (2019). Posterior nerve-sparing multilevel cervical corpectomy and reconstruction for metastatic cervical spine tumors: case report and literature review. *World Neurosurgery*.

[18] Miao D. C., Zhang B. Y., Lei T., Shen Y. (2017). Clinical efficacy of anterior partial corpectomy and titanium mesh fusion and internal fixation for treatment of old fracture dislocation of the lower cervical spine. *Medical Science Monitor*.

[19] Yan C., Jia H. C., Tan H. Y. (2021). How much space of the spinal canal should be restored by hoisting the vertebrae-opll complex for sufficient decompression in anterior controllable antedisplacement and fusion? A multicenter clinical radiological study. *The Spine Journal*.

[20] Park J. B., Yang J. H., Chang D. G. (2020). Comparison of union rates between autogenous iliac crest bone graft and local bone graft as fusion materials in lumbar fusion surgery: an evaluation of up to 3-level fusion. *World Neurosurgery*.

[21] Hatanaka H., Takasaki M., Furusho H., Omori Y. (2018). Cylinder-shaped bone graft for scaphoid nonunion. *The Journal of Hand Surgery (Asian-Pacific Volume)*.

[22] Islam M. M., Shahruzzaman M., Biswas S., Nurus Sakib M., Rashid T. U. (2020). Chitosan based bioactive materials in tissue engineering applications-a review. *Bioactive Materials*.

[23] Chen G., Xin B., Yin M. (2019). Biomechanical analysis of a novel height-adjustable nano-hydroxyapatite/polyamide-66 vertebral body: a finite element study. *Journal of Orthopaedic Surgery and Research*.

[24] Li Y. L., Zhao W. K., Zhang J. (2020). In vitro and in vivo evaluations of nano-hydroxyapatite/polyamide 66/yttria-stabilized zirconia as a novel bioactive material for bone screws: biocompatibility and bioactivity. *Journal of Biomaterials Applications*.

[25] Chen G., Yin M., Liu W. (2019). A novel height-adjustable nano-hydroxyapatite/polyamide-66 vertebral body for reconstruction of thoracolumbar structural stability after spinal tumor resection. *World Neurosurgery*.

[26] Yang X., Song Y., Liu L. (2014). Effectiveness of nano-hydroxyapatite/polyamide 66 cage in anterior spinal reconstruction: a mid-term study. *Zhonghua Wai Ke Za Zhi*.

